The article "Long non-coding RNA PVT1 promotes tumor progression by regulating the miR-143/HK2 axis in gallbladder cancer" was retracted in 2025. Reasons: duplicated data; duplicate publication; overlap with earlier publications; unreliable data.

# Long non-coding RNA PVT1 promotes tumor progression by regulating the miR-143/HK2 axis in gallbladder cancer

**DOI:** 10.1186/s12943-019-0947-9

**Published:** 2019-03-02

**Authors:** Jianan Chen, Yan Yu, Hua Li, Qiuyue Hu, Xiaolong Chen, Yuting He, Chen Xue, Fang Ren, Zhigang Ren, Juan Li, Liwen Liu, Zhenfeng Duan, Guangying Cui, Ranran Sun

**Affiliations:** 1 Precision Medicine Center, The First Affiliated Hospital of Zhengzhou University, Zhengzhou, 450052 China; 2 Key Laboratory of Clinical Medicine, The First Affiliated Hospital of Zhengzhou University, Zhengzhou, 450052 China; 3 Sarcoma Biology Laboratory, Department of Orthopaedic Surgery, David Geffen School of Medicine at University of California Los Angeles, Los Angeles, CA 90095 USA; 4 National Engineering Laboratory for Internet Medical System and Application, The First Affiliated Hospital of Zhengzhou University, Zhengzhou, 450052 Henan China

**Keywords:** Long non-coding RNA, PVT1, HK2, miR-143, Gallbladder cancer

## Abstract

**Background:**

The long non-coding RNA PVT1 (lncRNA PVT1) has been reported to act as an oncogenic regulator of several cancers. However, its expression and function in gallbladder cancer (GBC) remain largely unknown.

**Methods:**

In situ hybridization (ISH) and quantitative real-time PCR (qPCR) were performed to detect the expression of PVT1 and miR-143 in GBC tissues and cell lines. Immunohistochemistry (IHC) assays were performed to assess the expression of the hexokinase 2 (HK2) protein. The relationships among PVT1, miR-143 and HK2 were evaluated using dual-luciferase reporter, RNA immunoprecipitation (RIP) and biotin pull-down assays. The biological functions of PVT1, miR-143 and HK2 in GBC cells were explored with cell counting kit 8 (CCK-8), 5-ethynyl-20-deoxyuridine (EdU), colony formation, transwell, wound healing and glucose metabolism assays in vitro. For in vivo experiments, a xenograft model was used to investigate the effects of PVT1 and HK2 on GBC.

**Results:**

PVT1 was upregulated in GBC tissues and cells and was positively associated with malignancies and worse overall survival. PVT1 knockdown inhibited cell proliferation, migration, and invasion in vitro and restrained tumor growth in vivo. Further studies demonstrated that PVT1 positively regulated HK2 expression via its competing endogenous RNA (ceRNA) activity on miR-143. Additionally, HK2 expression and function were positively correlated with PVT1. Furthermore, we observed that the PVT1/miR-143/HK2 axis promoted cell proliferation and metastasis by regulating aerobic glucose metabolism in GBC cells.

**Conclusions:**

The results of our study reveal a potential ceRNA regulatory pathway in which PVT1 modulates HK2 expression by competitively binding to endogenous miR-143 in GBC cells, which may provide new insights into novel molecular therapeutic targets for GBC.

The article "Long non-coding RNA PVT1 promotes tumor progression by regulating the miR-143/HK2 axis in gallbladder cancer" was retracted in 2025. Reasons: duplicated data; duplicate publication; overlap with earlier publications; unreliable data.

**Electronic supplementary material:**

The online version of this article (10.1186/s12943-019-0947-9) contains supplementary material, which is available to authorized users.

## Background

Gallbladder cancer (GBC) is the most common and aggressive neoplasm of the biliary tract system [1]. The 5-year survival rate of GBC patients is less than 5% due to early metastasis, late diagnosis and poor prognosis [2, 3]. Currently, the complete surgical resection of GBC is the most efficient therapeutic method [4]. However, by the time most patients have been diagnosed with GBC, the optimal time for operation has passed. Therefore, it is of paramount importance to identify efficient prognostic biomarkers and therapeutic targets for GBC.

Long non-coding RNAs (lncRNAs) are a class of non-coding RNA that are at least 200 nucleotides in length and without protein-coding potential [5]. Numerous studies have demonstrated that lncRNAs frequently exhibit dysregulated expression in cancers and play critical roles in tumor initiation and progression [6–8]. The lncRNA plasmacytoma variant translocation 1 (PVT1) is located on chromosome 8q24, a region containing the well-accepted oncogene c-myc [9, 10]. Previous studies have shown that PVT1 acts as an oncogenic molecule in multiple human cancers, including breast cancer [11], gastric cancer [12] and colorectal cancer [13]. However, the functions and mechanisms of PVT1 with respect to GBC are still unclear.

Notably, lncRNAs, including PVT1, are well acknowledged to function as competing endogenous RNAs (ceRNAs) that can influence mRNA or other lncRNA transcripts by competitively binding to miRNA response elements (MREs) to modulate cancer-related gene expression. For example, PVT1 can promote the metastasis and proliferation of colon cancer by suppressing miR-30d-5p [14]. PVT1 has also been shown to promote epithelial to mesenchymal transition (EMT) and tumor development by interacting with miRNA-186 in prostate cancer cells [15]. However, whether PVT1 affects the biological behavior of GBC cells by regulating miRNAs has not been determined. Therefore, in this study, we focus on investigating the interaction between PVT1 and miRNAs in GBC cells. We report that a novel regulatory pathway composed of PVT1/miR-143/HK2 is involved in the progression of GBC, providing a potential biomarker and therapeutic target for GBC diagnosis and therapy.

## Methods

### Patients and specimens

The cohorts of GBC patients used in this study were described previously and contained fifty-three GBC tissues and 27 adjacent non-tumorous tissues from the First Affiliated Hospital of Zhengzhou University (Zhengzhou, China) as well as 79 GBC tissues and 20 adjacent normal tissues from Outdo Biotech (Shanghai, China) [16]. The clinicopathologic features of these patients are presented in Table 1. The study was approved by the Institutional Review Board of the First Affiliated Hospital of Zhengzhou University, and informed consent was obtained from all patients.

The article "Long non-coding RNA PVT1 promotes tumor progression by regulating the miR-143/HK2 axis in gallbladder cancer" was retracted in 2025. Reasons: duplicated data; duplicate publication; overlap with earlier publications; unreliable data.

**Table 1:** The relationship between PVT1 expression status and clinic-pathologic features of gallbladder cancer

	Clinicopathological features	No. of cases(*n*)	PVT1 expression		P	HK2 expression		P
			High(n = 33)	Low(*n* = 33)		High(*n* = 30)	Low(*n* = 36)	
Age(years)	<median	33	17	16	0.806	14	19	0.825
	>median	33	16	17		16	17	
Gender	Male	19	10	9	0.786	7	12	0.341
	Female	47	23	24		23	24	
Tumor size	< 5 cm	35	17	18	0.805	15	20	0.874
	> 5 cm	31	16	15		15	16	
TNM stage	Stage I and II	31	11	20	0.026^*^	9	22	0.042^*^
	Stage III and IV	35	22	13		21	14	
Distant metastasis	Absent	37	16	21	0.215	12	25	0.033^*^
	Present	29	17	12		18	11	
Differentiation grade	Stage I and II	28	11	17	0.135	8	20	0.004^*^
	Stage III and IV	38	22	16		22	16	

Abbreviations: TNM = tumor-node-metastasis; PVT1 = plasmacytoma variant translocation 1; HK2 = Hexokinase 2; ^*^P < .05

### Cell lines and culture

The human gallbladder cancer cell lines (GBC-SD and NOZ) and the human gallbladder epithelium cell line H69 used in this study were obtained from the Cell Bank of the Chinese Academy of Science (Shanghai, China). Cells were maintained in Dulbecco’s modified Eagle’s medium (DMEM) supplemented with 10% fetal bovine serum (FBS) (Gibco, NY, USA) and 100 U/ml penicillin/streptomycin (Corning, NY, USA) in a humidified incubator under a 5% CO_2_ atmosphere at 37 °C. All of the cell lines used in this study had been passed for less than 6 months in culture when the experiments were performed.

### Quantitative real-time PCR (qPCR)

Total RNA was extracted from GBC tissues and cells by using TRIzol reagent (Invitrogen, CA, USA) following the manufacturer’s instructions. The miRNAs and lncRNAs were reverse transcribed by using PrimeScript RT Master Mix (Takara, Dalian, China) following the manufacturer’s protocol. The relative quantification of PVT1 was performed using the 2^-△△Ct^ method, with β-actin used as an internal control. MiR-143 expression was normalized to the internal control U6 using the 2^-△△Ct^ method. The reactions were performed independently in triplicate, and the primer sequences are listed in Additional file 1: Table S1.

### Oligonucleotides and transfection

Three PVT1-specific siRNAs (si-PVT1–1, si-PVT1–2 and si-PVT1–3) were used to knock down PVT1, and a non-silencing siRNA (si-NC) oligonucleotide was used as a negative control (GenePharma, Shanghai, China). The cDNA encoding PVT1 was PCR amplified and then subcloned into the vector pcDNA3.1 (Invitrogen, CA, USA), generating the vector pcDNA-PVT1. The empty pcDNA3.1 vector (pcDNA-NC) was used as a control. The miR-143 mimics, inhibitor, HK2 siRNA (si-HK2) and the corresponding negative controls were synthesized by GenePharma. For transfections, 1 × 10^6^ cells (per well) were plated into a six-well plate, and plasmids were transfected into the cells using Lipofectamine 2000 (Invitrogen, CA, USA) following the manufacturer’s protocol. The transfected cells were harvested after 48 to 72 h. The transfection efficiency was determined by qPCR, and the PVT1-specific siRNA sequences are listed in Additional file 2: Table S2.

The article "Long non-coding RNA PVT1 promotes tumor progression by regulating the miR-143/HK2 axis in gallbladder cancer" was retracted in 2025. Reasons: duplicated data; duplicate publication; overlap with earlier publications; unreliable data.

### Generation of stable cell lines with overexpression or downregulation of PVT1

For the stable knockdown of PVT1, the most effective siRNA sequences were subcloned into the LV-12 (pGLVH6-CMV-LUC-2A-Puro-U6-shRNA) vector to generate a PVT1-shRNA lentivirus (lenti-sh-PVT1) (GenePharma). GBC-SD and NOZ cells were infected with the concentrated virus. For overexpression of PVT1, the PVT1 cDNA was PCR amplified and subcloned into the LV-13 (pLenti-EF1a-LUC-F2A-Puro-CMV) vector (GenePharma), and GBC-SD cells were infected with the concentrated virus. Subsequently, cells were treated with 2 μg/ml puromycin for 2 weeks to select for stable cell lines, in which the expression of PVT1 was validated by qPCR analysis.

### Tumor xenograft experiments

Female BALB/c nude mice (4 weeks old) were obtained from Vital River Laboratory Technology (Beijing, China) and housed and maintained in laminar airflow cabinets under specific pathogen-free conditions. Subsequently, the stable lenti-sh-PVT1 or lenti-PVT1 constructs and lenti-sh-HK2 GBC-SD or control cells (1 × 10^7^ cells/mice in 200 μl PBS) were injected subcutaneously into BALB/C nude mice. Tumor growth was measured after 1 week, and tumor volumes were calculated by the formula: volume (cm^3^) = (length × width^2^) / 2. After 4 weeks, the mice were sacrificed and the tumors were collected and weighed. All procedures were conducted in accordance with the Guidelines for the Care and Use of Laboratory Animals with the approval of the Ethics Committee of the First Affiliated Hospital of Zhengzhou University.

### Cell growth assay

For cell growth assays, 5 × 10^3^ cells per well were seeded into 96-well plates, with three wells used for each assayed group. Cell numbers were evaluated over 5 days using a cell counting kit-8 (CCK-8) (Dojindo, Kyushu, Japan). Ten microliters of CCK-8 reagent was added to each well, after which the plate was incubated at 37 °C for 2 h. Subsequently, the absorbance at 450 nm was measured in each well by using a spectrophotometer (Molecular Devices, CA, USA). The DNA synthesis rate was assayed by using a 5-ethynyl-20-deoxyuridine (EdU) assay kit (Ribobio, Guangzhou, China) following the manufacturer’s instructions. Images were taken and analyzed with a microscope (Olympus, Tokyo, Japan) at 100× magnification. The ratio of EdU-stained cells (with red fluorescence) to Hoechst-stained cells (with blue fluorescence) was used to evaluate the cell proliferation activity. For the colony formation assay, 1000 cells/well were plated into 6-well plates and routinely cultured for 14 days. The cells were subsequently fixed with 30% formaldehyde for 15 min and stained with 0.1% crystal violet. The number of colonies (containing more than 50 cells) was determined under an optical microscope.

The article "Long non-coding RNA PVT1 promotes tumor progression by regulating the miR-143/HK2 axis in gallbladder cancer" was retracted in 2025. Reasons: duplicated data; duplicate publication; overlap with earlier publications; unreliable data.

### Three-dimensional cell culture assay

To approximately mimic the in vivo environment, we conducted a three-dimensional (3D) cell culture assay to evaluate GBC cells growth and proliferation after HK2 depletion. In brief, after transfection with si-HK2 for 48 h, cells were plated in a Perfecta3D 96-well Hanging Drop plate (3D Biomatrix, NJ, USA). After incubating for 1 week at 37 °C, the cells were visualized and imaged.

### Cell migration and invasion assays

Cell migration was evaluated using a wound healing assay as described previously [17]. Briefly, cells were seeded into triplicate wells of a 6-well plate and were cultured to 30–50% confluence, after which artificial scratches were formed using a 20 μl pipette tip. The cell layers were imaged, and migration was monitored at 0 and 48 h after scratching using an Olympus 1X71 camera system. The invasive ability of the cells was accessed using a transwell assay. Cells (5 × 10^4^) were seeded onto a transwell plate with 8-mm pores, and DMEM supplemented with 20% FBS was used as a chemoattractant. Following a 24-h incubation, non-invading cells were manually removed using a cotton swab. Subsequently, the cells were fixed in 4% paraformaldehyde for 20 min, stained with haematoxylin and then counted under a microscope.

### Glucose consumption and lactic acid assays

Glucose consumption was quantified by glucose oxidase-peroxidase (Sigma, MO, USA) reaction coupled with oxidation of Amplex Red reagent (Life Technologies, CA, USA) according to the manufacturer’s protocol. Glucose consumption was calculated by subtracting the amount of glucose present in cell culture medium without any cells. Lactic acid produced in the medium was quantified using a lactic acid assay kit (Sigma, MO, USA) according to the manufacturer’s protocol. The OD value was measured and applied to the standard curve to calculate the test samples.

The article "Long non-coding RNA PVT1 promotes tumor progression by regulating the miR-143/HK2 axis in gallbladder cancer" was retracted in 2025. Reasons: duplicated data; duplicate publication; overlap with earlier publications; unreliable data.

### Glycolysis stress test

Extracellular acidification rate (ECAR) and oxygen consumption rate (OCR) analyses were conducted to evaluate the effect of PVT1 depletion on glycolysis stress and cell mitochondrial stress using the Seahorse XF96 Glycolysis Analyzer (Seahorse Bioscience, MA, USA). For ECAR analysis, glucose, oligomycin, and 2-deoxyglucose were sequentially added in special medium. Glucose was first injected into the medium and catabolized to lactate and ATP with a corresponding increased ECAR value. Then, oligomycin was injected, which inhibited mitochondrial ATP production and shifted the energy production to glycolysis, with the corresponding increase in ECAR. The ECAR was reported in milli-pH (mpH) units per minute.

For OCR analysis, first the ATP synthase inhibitor oligomycin was injected into the medium, and the induced decrease in OCR was associated with the proton current resulting from ATP synthase. Carbonyl cyanide 4-(trifluoromethoxy) phenylhydrazone (FCCP) was then injected, leading to rapid oxygen consumption. Compared with basal respiration, the induced increased respiratory capacity indicated the spare respiratory capacity. Finally, rotenone and antimycin A, electron transport chain inhibitors, were injected. Residual respiration corresponds to the non-mitochondrial respiration. The OCR was reported in units of picomoles per minute.

### Western blotting

Western blotting was performed as described previously [17]. Briefly, cells were collected and lysed using RIPA protein extraction reagent (Beyotime) with a protease inhibitor cocktail (Roche, IN, USA). Equal amounts of protein were electrophoresed on 10% SDS-PAGE gels and then transferred to polyvinylidene difluoride (PVDF) membranes (Millipore, MA, USA), which were then blocked in buffer (5% free-fat milk in TBST) before being incubated with the anti-rabbit HK2, CDK4, CDK6, PCNA, MMP-2 and MMP-9 antibodies (1:1000 dilution, Proteintech) and anti-rabbit Ki-67 antibody (1:1000 dilution, Signalway Antibody, TX, USA) at 4 °C for 12 h. Anti-mouse β-actin antibody (1:5000 dilution, Proteintech) was used as a loading control. Horseradish peroxidase-conjugated goat anti-rabbit or goat anti-mouse IgG antibody (1:5000, Beyotime) was applied as a secondary antibody.

### Immunohistochemical (IHC) staining and in situ hybridization (ISH)

IHC staining was performed according to our previous study. Briefly, TMA sections were deparaffinized and rehydrated, and antigen retrieval was conducted with Target Retrieval Solution (Dako, CA, USA) following the manufacturer’s instructions. Endogenous peroxidase activity was blocked with 0.3% hydrogen peroxide for 15 min. Slides were then blocked with goat serum, avidin solution and biotin solution. The slides were incubated with rabbit anti-human polyclonal antibodies against HK2 (1:200 dilution, Proteintech) and Ki-67 (1:500 dilution, Signalway Antibody) at 4 °C overnight and then probed with biotinylated goat anti-rabbit secondary antibody (Vector Laboratories, CA, USA) and high-sensitivity streptavidin–HRP conjugate. To visualize staining, slides were incubated in 3, 30-diaminobenzidine in 0.1% H_2_O_2_ in Tris–HCl buffer and subsequently counterstained with Hematoxylin QS (Vector Laboratories).

The article "Long non-coding RNA PVT1 promotes tumor progression by regulating the miR-143/HK2 axis in gallbladder cancer" was retracted in 2025. Reasons: duplicated data; duplicate publication; overlap with earlier publications; unreliable data.

Expression of PVT1 in GBC was detected using biotin-labeled PVT1 ISH probes (BOSTER, Wuhan, China) for TMA on the basis of the protocol provided by the manufacturer. Briefly, TMA slides were fixed in 4% paraformaldehyde and then incubated with proteinase-K for 20 min at 37 °C. The slides were hybridized with PVT1 probe (200 nM) for 40 min at 50 °C. The slides were incubated with anti-DIG reagent, and the probe signal was visualized with diaminobenzidine (DAB) solution (BOSTER). Two pathologists evaluated the IHC and ISH scores in a blinded manner. The intensity of PVT1 or HK2 staining was scored on a scale of 1–4 as follows: 1 (no staining), 2 (weak staining), 3 (moderate staining) and 4 (strong staining). Tissues with scores of 3 and 4 were defined as high expression group, and those with scores of 1 and 2 were classified as exhibiting low expression.

### Luciferase reporter assay

Bioinformatics tools (microRNA.org) were used to predict the miR-143 binding sites of PVT1. Human GBC-SD cells were transfected with 150 ng of empty pmirGLO-NC, pmirGLO-PVT1-wt or pmirGLO-PVT1-mut (GenePharma). Two nanograms of pRL-TK (Promega, WI, USA) were cotransfected with the miR-143 mimic or miR-NC into GBC-SD cells by using Lipofectamine 2000 (Invitrogen) following the manufacturer’s procedures. The relative luciferase activity was normalized to Renilla luciferase activity 48 h after transfection.

### RNA immunoprecipitation (RIP) assay

The RIP assay was conducted by using a Thermo Fisher RIP kit (Thermo Fisher Scientific, MA, USA) following the manufacturer’s instructions. Briefly, cells were lysed in RIP lysis buffer, and RNAs magnetic beads were conjugated with a human anti-AGO2 antibody or with a negative control normal mouse anti-IgG. Subsequently, the retrieved RNA was assayed by qPCR.

### RNA pull-down assay

A DNA fragment containing the full-length PVT1 sequence or a negative control sequence was PCR amplified using T7 RNA polymerase (Roche, Basel, Switzerland). The resulting plasmid DNA was linearized using the restriction enzyme *Xho*I. Biotin-labeled RNA was reverse transcribed using Biotin RNA Labeling Mix (Roche) and T7 RNA polymerase (Takara Biomedical Technology). The products were treated with RNase-free DNase I (Roche) and purified with an RNeasy Mini Kit (Qiagen, MD, USA), with the resulting RNA used for real-time PCR assays.

The article "Long non-coding RNA PVT1 promotes tumor progression by regulating the miR-143/HK2 axis in gallbladder cancer" was retracted in 2025. Reasons: duplicated data; duplicate publication; overlap with earlier publications; unreliable data.

### RNA-FISH and subcellular fractionation of PVT1

Cy3-labeled PVT1 and DAPI-labeled U6 probes were obtained from RiboBio (Guangzhou, China). RNA fluorescence in situ hybridization (FISH) was performed using a FISH kit (RiboBio) following the manufacturer’s instructions. A nucleus and cytoplasm segmentation PARIS™ kit (Ambion, TX, USA) was used to segment the nucleus and cytoplasm of cells following the manufacturer’s instructions.

### Collection of GBC microarray data

Microarray datasets (GSE76633 and GSE104165) available online were assembled using the Gene Expression Omnibus (GEO) of the National Center for Biotechnology Information (NCBI). The BRB-array tools were used to identify the differentially expressed genes between healthy or adjacent non-tumorous tissues and GBC. For the GSE104165 dataset, R language was utilized to screen out the differentially expressed microRNAs according to the criteria “adjusted P < 0.05 (FDR 0.05) and |fold change| > 2.” After the sequences were sorted by fold change and *P* values, the top 10 downregulated miRNAs were selected to generate a heatmap with R language.

### Statistical analysis

All experiments were performed in triplicate. Statistical analyses were performed using SPSS (version 23.0, SPSS Inc.) or GraphPad Prism software (version 7.0, USA). Clinicopathological characteristics were analyzed by chi-square tests. Survival curves were generated using the Kaplan-Meier method and log-rank tests. Univariate and multivariate Cox regression analyses were conducted to identify the independent factors. Student’s t-test or the Mann–Whitney U test was used for comparison between two groups depending on distribution. *P* (two-sided) less than 0.05 was considered to indicate statistical significance. All data were presented as the mean ± standard deviation (SD).

## Results

### PVT1 expression is upregulated in GBC tissues

Analysis of the GSE76633 dataset from the GEO database revealed that the expression of PVT1 was significantly upregulated in GBC tissues (Fig. 1a). To confirm this result, we assessed PVT1 expression in 20 GBC tissues and their corresponding adjacent non-tumorous tissues. The qPCR analysis data showed that PVT1 was overexpressed in GBC tissues (Fig. 1b). Additionally, we examined PVT1 expression in 121 cancerous and 41 peritumoral tissues from GBC patients using ISH. As shown in Fig. 1c, GBC specimens exhibited various degrees of PVT1 expression, with staining primarily observed in the cell cytoplasm. PVT1 expression was elevated in most tumor tissues compared to non-tumor tissues (Fig. 1d and e). High PVT1 expression was associated with advanced tumor-node-metastasis (TNM) stage and distant metastasis (Fig. 1e). A detailed summary of the relationships between PVT1 expression and the clinicopathologic features of GBC patients is provided in Table 1. Importantly, with regard to overall survival (OS), PVT1 overexpression correlated with worse OS rate (Fig. 1f). Additionally, univariate and multivariate analyses showed that PVT1 was a potent independent prognostic indicator for GBC patients apart from TNM stage (Table 2). These results indicated that the upregulation of PVT1 might play an important role in GBC progression.

The article "Long non-coding RNA PVT1 promotes tumor progression by regulating the miR-143/HK2 axis in gallbladder cancer" was retracted in 2025. Reasons: duplicated data; duplicate publication; overlap with earlier publications; unreliable data.

**Fig. 1:** PVT1 is significantly upregulated in GBC tissues and cell lines. **(a)** PVT1 expression levels in GBC tissues and paired non-tumor tissues of the GEO database (GSE76633). **(b)** PVT1 was upregulated in GBC tissues detected by qPCR in 20 pairs of GBC tissues. **(c)** Representative PVT1 staining patterns. Scale bar, 100 μm. (d**-e)** The expression level of PVT1 was higher in GBC tissues than adjacent normal tissues. Scale bar, 100 μm. High PVT1 expression correlated with advanced TNM stage and distant metastasis. **(f)** High PVT1 expression was significantly associated with poor OS in GBC patients. *P < 0.05, **P < 0.01, ***P < 0.001. Error bars indicate mean ± SD

**Table 2:** Univariate and multivariate analyses of overall survival of gallbladder cancer

	Clinicopathological parameters	Overall survival (OS)		
		HR	95%(CI)	*P* value
Univariate analyses	Age (>median vs. ≤median)	1.102	0.607–1.998	0.750
	Gender (male vs. female)	1.289	0.663–2.507	0.454
	Tumor size (> 5 cm vs. ≤5 cm)	1.199	0.664–2.168	0.547
	TNM stage (III-IV vs. I-II)	4.525	2.296–8.919	< 0.001**
	Distant metastasis (Present vs. Absent)	2.894	1.448–5.783	0.003**
	PVT1 expression (High vs. Low)	2.467	1.338–4.548	0.004**
	HK2 expression (High vs. Low)	2.220	1.246–3.953	0.007**
Multivariate analyses	TNM stage (III-IV vs. I-II)	4.119	2.061–8.232	< 0.001**
	Distant metastasis (Present vs. Absent)	2.059	1.010–4.196	0.047**
	PVT1 expression (High vs. Low)	1.986	1.055–3.739	0.033**
Multivariate analyses	TNM stage (III-IV vs. I-II)	2.444	1.267–4.714	0.008**
	Distant metastasis (Present vs. Absent)	1.936	1.024–3.469	0.041**
	HK2 expression (High vs. Low)	1.842	1.103–3.351	0.045**

Abbreviations: TNM = tumor-node-metastasis; HR = hazard ratio; CI = confidential interval; PVT1 = plasmacytoma variant translocation 1; HK2 = Hexokinase 2; **P < .05

The article "Long non-coding RNA PVT1 promotes tumor progression by regulating the miR-143/HK2 axis in gallbladder cancer" was retracted in 2025. Reasons: duplicated data; duplicate publication; overlap with earlier publications; unreliable data.

### Knockdown of PVT1 inhibits GBC cell proliferation, migration and invasion in vitro

To further explore the biological role of PVT1 in GBC, we first examined the level of PVT1 in GBC cell lines and observed that PVT1 was highly expressed in GBC cell lines compared with normal H69 cells (Additional file 3: Fig. S1a). The nucleus and cytoplasm segmentation and RNA-FISH analyses confirmed that PVT1 was localized predominantly in the cell cytoplasm rather than the nucleus, indicating that PVT1 primarily exerted an effect on GBC in the cytoplasm (Additional file 3: Fig. S1b-d). We next transfected GBC-SD and NOZ cells with PVT1-siRNAs (si-PVT1–1, si-PVT1–2 and si-PVT1–3) and the negative control (si-NC). The transfection efficiency was confirmed by qPCR (Fig. 2a and b). Next, si-PVT1–1 and si-PVT1–3 were selected for further experiments on the basis of their more effective inhibition. Subsequently, the results of the CCK-8 assay demonstrated that the PVT1 knockdown significantly inhibited cell proliferation (Fig. 2c and d). In parallel, the colony formation assay showed significantly lower colony numbers after PVT1 depletion (Fig. 2e and f). The EdU assay demonstrated that suppression of PVT1 attenuated the proliferation of GBC cells (Fig. 2g and h). Moreover, we observed that cell invasion and migration were suppressed in GBC cells transfected with si-PVT1 compared with cells transfected with si-NC using transwell and wound healing assays (Fig. 2i-l). Consistent with the above findings, PVT1 knockdown remarkably decreased the expression of the cell proliferation proteins Ki-67 and PCNA as well as the G1/S-phase checkpoint protein CDK4 but not CDK6 (Additional file 4: Figure S2a and 2b). In addition, PVT1 knockdown significantly inhibited the expression of two matrix metalloproteinases, MMP-2 and MMP-9, which were closely associated with metastasis (Additional file 4: Figure S2c and 2d). Furthermore, by analyzing the GSE76633 dataset, we validated the correlation between PVT1 and these proteins (Additional file 4: Figure S2e and 2f). These results indicated the potential carcinogenicity of PVT1 in GBC.

**Fig. 2:** The effect of PVT1 on GBC cells biological behavior in vitro. **(a-b)** PVT1 expression was knocked down by three siRNAs targeting PVT1 in GBC-SD and NOZ cells. **(c-d)** Knockdown of PVT1 significantly decreased cell proliferation compared with si-NC cells using CCK-8 assay. **(e-f)** Colony numbers of GBC-SD and NOZ cells transfected with si-PVT1 were significantly lower than in those transfected with si-NC. **(g-h)** EdU assay showed that suppression of PVT1 attenuated the proliferation of GBC-SD and NOZ cells (magnification, × 100). Scale bar, 100 μm. (**i**-**l**) PVT1 suppression impaired GBC cell invasion and migration, as measured by a transwell assay (magnification, × 100). Scale bar, 100 μm and wound healing assay, respectively. *P < 0.05, **P < 0.01, ***P < 0.001. Error bars indicate mean ± SD

The article "Long non-coding RNA PVT1 promotes tumor progression by regulating the miR-143/HK2 axis in gallbladder cancer" was retracted in 2025. Reasons: duplicated data; duplicate publication; overlap with earlier publications; unreliable data.

### PVT1 binds to miR-143 and suppresses its expression

To identify the potential mechanisms by which PVT1 functioned in GBC cells, we used an online bioinformatics database (DIANA) to predict the potential targets for PVT1, the detailed results of which are displayed in Additional file 5: Table S3. Furthermore, we extracted and analyzed the GSE104165 cohort from the GEO database. The results revealed that miR-143, a significant tumor suppressor in GBC [18], had putative PVT1 binding sites (Fig. 3a) and was one of the most downregulated miRNAs in GBC tissues (Additional file 6: Table S4 and Additional file 7: Figure S3). The qPCR data showed that miR-143 was downregulated in 20 pairs of GBC tissues, and a negative correlation between PVT1 and miR-143 expression was observed (Fig. 3b and c). Moreover, knockdown of PVT1 significantly increased miR-143 expression, while GBC cells transfected with pcDNA-PVT1 upregulated PVT1 expression and exhibited a dramatic inhibition of miR-143 expression (Fig. 3d-f).

**Fig. 3:** PVT1 negatively regulates miR-143 expression. **(a)** The potential binding sites between miR-143 and PVT1. **(b-c)** miR-143 was downregulated in GBC tissues, and PVT1 expression and miR-143 expression were inversely correlated in GBC tissues. **(d)** MiR-143 expression was increased after PVT1 knockdown. **(e-f)** GBC-SD and NOZ cells were transfected with pcDNA-NC or pcDNA-PVT1. qPCR showed that pcDNA-PVT1 upregulated PVT1 expression and decreased miR-143 expression. **(g-h)** The expression level of PVT1 was decreased after transfection with miR-143 mimics but increased after transfection with miR-143 inhibitor. **(i)** Co-transfection of miR-143 mimics and pmirGLO-PVT1-wt strongly decreased the luciferase activity, while co-transfection of miR-143 mimics and pmirGLO-PVT1-mut did not change the luciferase activity. *P < 0.05, **P < 0.01, ***P < 0.001. Error bars indicate mean ± SD

Intriguingly, knockdown or overexpression of miR-143 could also affect PVT1 expression (Fig. 3g and h). We then performed luciferase reporter assay to validate the binding of miR-143 with PVT1. The results demonstrated that miR-143 overexpression remarkably reduced the luciferase activity of pmirGLO-PVT1-wt but not pmirGLO-PVT1-mut (Fig. 3i). In addition, the RIP assay results further confirmed that miR-143 was a target of PVT1 in GBC cells (Additional file 8: Figure S4a-d). Subsequently, the biotin-labeled pull-down results showed a significant amount of PVT1 and miR-143 in the PVT1 pull-down pellet compared with that observed in the control group as measured by qPCR (Additional file 8: Figure S4e and 4f). These data suggested that PVT1 could negatively regulate miR-143 expression in GBC cells.

The article "Long non-coding RNA PVT1 promotes tumor progression by regulating the miR-143/HK2 axis in gallbladder cancer" was retracted in 2025. Reasons: duplicated data; duplicate publication; overlap with earlier publications; unreliable data.

### PVT1 plays a ceRNA role in regulating HK2 expression by sponging miR-143

HK2 is a well-accepted oncogene targeted by miR-143 in tumors, such as colon cancer [19, 20]. Thus, we aimed to verify whether PVT1 could regulate HK2 expression by targeting miR-143 in GBC cells. Interestingly, the HK2 mRNA and protein levels in GBC-SD cells were significantly decreased after PVT1 knockdown but were upregulated when transfected with the miR-143 inhibitor. However, in the group co-transfected with si-PVT1 and the miR-143 inhibitor, the regulatory effects of PVT1 on HK2 expression were reversed (Fig. 4a and b). Additionally, the HK2 mRNA and protein levels were both increased in GBC-SD cells after PVT1 overexpression but were reversed by co-trasfection with pcDNA-PVT1 and miR-143 mimics (Fig. 4c and d). Moreover, as shown in Fig. 4e and f, the qPCR results showed that PVT1 was positively associated with HK2 mRNA transcript levels in the GSE76633 dataset or the same 20 pairs of GBC tissues. The above results suggested that PVT1 regulated HK2 expression by sponging miR-143.

**Fig. 4:** PVT1 regulates HK2 expression by sponging miR-143. **(a-b)** The effects of si-PVT1, miR-143 inhibitor and si-PVT1 + miR-143 inhibitor on mRNA and protein levels of HK2 in GBC-SD cells. **(c-d)** The effects of miR-143 mimics, pcDNA-PVT1, and miR-143 mimics+pcDNA-PVT1 on mRNA and protein levels of HK2 in GBC-SD cells. **(e-f)** Pearson correlation between PVT1 and HK2 mRNA transcript level was measured in GSE76633 and 20 pairs of GBC tissues, respectively. **(g-h)** Expression level of HK2 was higher in GBC tissues than in normal tissues by IHC staining. Scale bar, 100 μm. **(i)** Representative HK2 staining patterns. Scale bar, 100 μm. **(j-k)** High PVT1 expression correlated with advanced TNM stage, metastasis and poor overall survival. **(l)** The association between PVT1 and HK2 expression. *P < 0.05, **P < 0.01, ***P < 0.001. Error bars indicate mean ± SD

### Knockdown of HK2 inhibits tumor cell proliferation, migration and invasion of GBC cells in vitro and GBC growth in vivo

To explore the biological function of HK2 in GBC cells, we first demonstrated that HK2 was upregulated in GBC specimens via immunohistochemistry analyses (Fig. 4g-i). High HK2 expression was significantly correlated with advanced TNM stage, the presence of metastasis and poor prognosis (Fig. 4j and k). Moreover, there was a notable positive correlation between PVT1 and HK2 levels (Fig. 4l). The detailed information on HK2 expression and clinicopathologic parameters is shown in Table 1. Univariate analyses for OS revealed the HK2 level, distant metastasis, and TNM stage to be significant prognostic variables in GBC, and subsequent multivariate analysis showed that HK2 expression was an independent prognostic factor for GBC patients apart from the TNM stage (Table 2). We next used HK2-siRNA (si-HK2) and its negative control (si-ctrl) to transfect GBC-SD and NOZ cells, and the transfection efficiency was assessed by western blotting (Fig. 5a). Proliferation assays showed that downregulated HK2 significantly attenuated the GBC cell proliferation rate (Fig. 5b-e). Next, we conducted a three-dimensional cell culture assay to verify the above results in a mimicked in vivo environment, the results of which showed that the cancer spheroids formed from GBC-SD cells with HK2 inhibition were significantly smaller than those of the control group (Fig. 5f). Furthermore, transwell and wound healing assays demonstrated that the abilities of cell invasion and migration were significantly decreased in GBC cells transfected with si-HK2 compared to cells transfected with si-ctrl (Fig. 5g-i). Additionally, glucose consumption and cellular lactate production levels were remarkably reduced after HK2 knockdown (Fig. 5j and k). Furthermore, the results of in vivo experiments showed that HK2 knockdown inhibited the rate of GBC growth in xenograft models (Fig. 5l-o).

The article "Long non-coding RNA PVT1 promotes tumor progression by regulating the miR-143/HK2 axis in gallbladder cancer" was retracted in 2025. Reasons: duplicated data; duplicate publication; overlap with earlier publications; unreliable data.

**Fig. 5:** HK2 promotes cell proliferation, invasion and migration in vitro and tumor growth in vivo. **(a)** The protein levels of HK2 in GBC cells after knockdown by si-HK2. **(b-e)** Knockdown of HK2 significantly decreased cell proliferation compared with si-ctrl cells by proliferation assays. **(f)** Formation of spheres from GBC cells transfected with si-HK2 accessed by three-dimensional cell culture (magnification, × 200, scale bar, 50 μm). **(g-i)** HK2 suppression impaired GBC cell invasion and migration, as measured by transwell assay (magnification, × 100). Scale bar, 100 μm and wound healing assays. **(j-k)** Glucose consumption and lactate production were significantly decreased after HK2 knockdown. **(l-m)** Tumor volume and weight in the lenti-sh-HK2 group were significantly lower than those in the lenti-sh-NC group. **(n)** Images of tumor formation were performed by a live imaging system detecting the luciferase signal. **(o)** The luciferase activity in the lenti-sh-HK2 group was lower than that in the lenti-sh-NC group. *P < 0.05, **P < 0.01, ***P < 0.001. Error bars indicate mean ± SD

The article "Long non-coding RNA PVT1 promotes tumor progression by regulating the miR-143/HK2 axis in gallbladder cancer" was retracted in 2025. Reasons: duplicated data; duplicate publication; overlap with earlier publications; unreliable data.

### MiR-143 mimics reverse the oncogenic function of PVT1 in vitro

To determine whether PVT1 induced GBC cell proliferation, migration and invasion through the miR-143/HK2 axis, we ectopically expressed miR-143 in stable PVT1-overexpressed GBC-SD and NOZ cells. The results of CCK-8 assays showed that the overexpression of miR-143 attenuated the promoted effect of PVT1 on cell proliferation (Fig. 6a and b). Similar results were also observed in colony formation assays (Fig. 6c and d). In addition, the results of the transwell and wound healing assays revealed that miR-143 overexpression counteracted the effect of PVT1 in promoting cell invasion and migration (Fig. 6e-h). These results showed that PVT1 promoted tumor cell growth and metastasis at least in part via the miR-143/HK2 axis.

**Fig. 6:** MiR-143 mimics reverse the oncogenic function of PVT1 in vitro. **(a-b)** CCK-8 assay showed that the introduction of miR-143 mimics attenuated the proliferation-promoting effect of PVT1 in GBC cells. **(c-d)** The introduction of miR-143 mimics attenuated the colony formation-promoting effect of PVT1 in GBC cells. **(e-h)** The abilities of cell invasion and migration induced by PVT1 were significantly attenuated after the introduction of miR-143 mimics in GBC-SD and NOZ cells, as measured by transwell assay (magnification, × 100). Scale bar, 100 μm and wound healing assays. *P < 0.05, **P < 0.01, ***P < 0.001. Error bars indicate mean ± SD

### The PVT1/miR-143/HK2 axis regulates glucose metabolism in GBC cells

Given that HK2 functioned as a significant metabolic enzyme in glucose utilization, we were interested in assessing whether glucose metabolism was regulated by the PVT1/miR-143/HK2 axis in GBC cells. As shown in Fig. 7a and b, we noted an obvious decrease in glucose consumption and cellular lactate production levels during PVT1 depletion but a remarkable increase in cells transfected with the miR-143 inhibitor. In contrast, in the group co-transfected with si-PVT1 and the miR-143 inhibitor, the effects of PVT1 on glycolysis were diminished. In parallel, glucose consumption and cellular lactate production levels were significantly increased in cells overexpressing PVT1, but this effect was counteracted in cells co-transfected with PVT1 plasmids and miR-143 mimics (Fig. 7c and d).

**Fig. 7:** The PVT1/miR-143/HK2 axis regulates glucose metabolism in GBC cells. **(a-b)** The effects of si-PVT1, miR-143 inhibitor and si-PVT1 + miR-143 inhibitor on glucose consumption and cellular lactate production levels in GBC-SD cells. **(c-d)** The effects of miR-143 mimics, pcDNA-PVT1, and miR-143 mimics+pcDNA-PVT1 on glucose consumption and cellular lactate production levels in GBC-SD cells. **(e-f)** ECAR was detected by the Glycolysis Stress Test in GBC-SD cells after transfection with si-PVT1 or si-NC. **(g-h)** OCR was measured by the Cell Mito Stress Test in GBC-SD cells after transfection with si-PVT1 or si-NC. *P < 0.05, **P < 0.01, ***P < 0.001. Error bars indicate mean ± SD

To further explore whether PVT1 regulated glucose metabolism in GBC cells, the glycolysis flux was evaluated based on ECAR using the Seahorse assay. The results showed that ECAR was decreased after PVT1 knockdown (Fig. 7e and f). Mitochondrial respiration was detected by OCR measurements to assess changes in the level of OxPhos-dependent ATP generation in GBC cells. We observed that GBC cells transfected with si-PVT1 exhibited a higher basal mitochondrial OCR and maximal OCR (Fig. 7g and h). Taken together, these results indicated that PVT1 could promote glycolysis by modulating the miR-143/HK2 axis in GBC cells.

The article "Long non-coding RNA PVT1 promotes tumor progression by regulating the miR-143/HK2 axis in gallbladder cancer" was retracted in 2025. Reasons: duplicated data; duplicate publication; overlap with earlier publications; unreliable data.

### PVT1 promotes the growth rate of GBC in vivo

To determine the function of PVT1 with respect to the carcinogenesis of GBC in vivo, we first determined the PVT1 expression levels in stable GBC-SD and NOZ cells transfected with lenti-sh-PVT1 or lenti-PVT1 and their corresponding controls (Additional file 9: Figure S5a and 5b). Next, the stable GBC-SD cells were injected into BALB/c nude mice to construct a xenograft model. As expected, a significant decrease in both tumor volume and weight was detected in the lenti-sh-PVT1 group compared with those observed in the lenti-sh-NC group (Fig. 8a-d). Additionally, lower Ki-67 and HK2 expression was observed in the lenti-sh-PVT1 group than in the lenti-sh-NC group (Fig. 8e-g). In contrast, the tumors in the lenti-PVT1 group grew more rapidly and had higher Ki67 and HK2 expression than the group infected with control cells (Fig. 8h-n). Taken together, these results suggested that PVT1 significantly promoted tumor growth of GBC in vivo by upregulating HK2 expression.

**Fig. 8:** PVT1 promotes tumor growth in vivo. **(a)** Images of tumor formation were performed by a live imaging system detecting the luciferase signal. **(b)** The luciferase activity in the lenti-sh-PVT1 group was lower than in the lenti-sh-NC group. **(c-d)** The volumes and weight of lenti-sh-PVT1 cell-derived xenograft tumors were markedly lower than those of the lenti-sh-NC group. **(e-g)** Sections of xenograft tumors stained with hematoxylin and eosin (H&E) as well as immunohistochemical staining for HK2 and Ki-67 (magnification, × 200). Scale bar, 100 μm. **(h)** Representative images of tumor formation of the lenti-NC group and lenti-PVT1 group. **(i)** The luciferase activity in the lenti-PVT1 group was higher than that in the lenti-NC group. **(j-k)** The volumes and weight of lenti-PVT1 cell-derived xenograft tumors were markedly higher than those of the lenti-NC group. **(l-n)** The levels of Ki67 and HK2 were much higher after PVT1 overexpression (magnification, × 200). Scale bar, 100 μm. *P < 0.05, **P < 0.01, ***P < 0.001. Error bars indicate mean ± SD

The article "Long non-coding RNA PVT1 promotes tumor progression by regulating the miR-143/HK2 axis in gallbladder cancer" was retracted in 2025. Reasons: duplicated data; duplicate publication; overlap with earlier publications; unreliable data.

## Discussion

Recently, a great deal of evidence has shown that PVT1 plays an important role in tumor progression. For instance, upregulated PVT1 was demonstrated to be associated with advanced tumor stage and poor survival in colorectal cancer [21] and non-small cell lung cancer (NSCLC) [22]. The abnormal expression of PVT1 in pancreatic cancer (PDAC) was correlated with invasion and poor prognosis [23]. In our study, we demonstrated that PVT1 was upregulated in GBC tissues and cells. High PVT1 expression was shown to be positively associated with advanced TNM stage and poorer OS in patients with GBC. In addition, PVT1 knockdown significantly suppressed the proliferation, migration and invasion of GBC cells in vitro and repressed tumor growth in vivo. These results were consistent with those of previous studies and indicated that PVT1 functioned as an oncogene in GBC.

A growing body of evidence has demonstrated that lncRNAs can serve as a natural miRNA sponge and regulate their functions [24–28]. In GBC, a lncRNA in prognosis-associated gallbladder cancer (PAGBC) was observed to competitively bind to miR-133b and miR-511 to promote tumor progression and activate the AKT/mTOR pathway [29]. Taurine upregulated 1 (TUG1) was reported to promote GBC cell proliferation, metastasis and EMT progression by functioning as an miRNA sponge to abrogate the endogenous effect of miR-300 [30]. To identify the underlying molecular mechanism of PVT1 activity in GBC cells, bioinformatics analysis revealed that miR-143, which had been previously demonstrated to be a tumor suppressor in several types of cancers, including GBC, prostate cancer and pancreatic cancer [31–33], might have potential PVT1 binding sites. We observed a negative dual-regulation between miR-143 and PVT1 by qPCR. Furthermore, the results of luciferase reporter, RIP and biotin pull-down assays confirmed that miR-143 was a direct target of PVT1.

HK2 is known to be a key metabolic enzyme by promoting glucose uptake in cells and facilitating the Warburg effect [34]. HK2 upregulation has been observed in many types of cancer, promoting tumor growth, metastasis and glycolysis as well as being a target of miR-143 in several cancers [19, 20, 35]. Our findings also suggested that HK2 expression was significantly higher in GBC tissues and positively associated with malignancies and poor prognosis. Downregulation of HK2 significantly inhibited cell proliferation, migration and invasion in GBC cells. In addition, after HK2 knockdown, the glucose consumption and cellular lactate production levels in GBC cells were profoundly decreased, which agreed well with the results of previous studies. For example, Wolf et al. reported that HK2 was overexpressed in glioblastoma multiforme (GBM) tumors and was crucial for the Warburg effect [36]. In hepatocellular carcinoma (HCC) cells, overexpression of HK2 could induce tumor development by promoting glycolysis [37]. More importantly, we observed that PVT1 could positively regulate HK2 expression by inhibiting miR-143 expression both in vitro and in vivo. Overexpression of miR-143 could repress the proliferation and metastasis ability promoted by PVT1 in GBC cells. Furthermore, PVT1 positively modulated glucose metabolism by repressing miR-143 expression in GBC cells, which agreed with the findings of previous studies showing that PVT1 promoted glycolysis and osteosarcoma progression by regulating the miR-497/HK2 pathway [38].

The article "Long non-coding RNA PVT1 promotes tumor progression by regulating the miR-143/HK2 axis in gallbladder cancer" was retracted in 2025. Reasons: duplicated data; duplicate publication; overlap with earlier publications; unreliable data.

## Conclusions

In sum, our study demonstrates that PVT1 functions as an oncogenic lncRNA during GBC progression and reveals a novel ceRNA regulatory pathway in which PVT1 upregulates HK2 expression by sponging miR-143. Thus, PVT1 is potentially a novel therapeutic target for GBC patients.

## Additional file

Additional file 1: **Table S1.** Primer sequence used in this study (DOCX 13 kb)

Additional file 2: **Table S2.** siRNA sequences used in this study. (DOCX 12 kb)

Additional file 3: **Figure S1.** Expression and subcellular location of PVT1 in human GBC. cell lines. **(a)** PVT1 expression was significantly higher in GBC cellscompared with the human gallbladder epithelium cell line H69. **(b-c)** nucleus and cytoplasm segmentation assay to determine the PVT1 expression in GBC-SD cells and NOZ cells. **(d)** Localization of PVT1 by RNA-FISH in GBC-SD and NOZ cells. Nuclei are stained blue (DAPI) and PVT1 is stained red (magnification, × 200, scale bar, 50 μm). *P < 0.05, **P < 0.01, ***P < 0.001. Error bars indicate mean ± SD. (PDF 197 kb)

Additional file 4: **Figure S2.** The related protein levels of cell proliferation, migration and invasion were reduced after PVT1 knockdown. **(a-b)** The protein expression of CDK4, CDK6, Ki-67, and PCNA was examined by western blot, and the relative protein expression was shown in histogram normalized to β-actin. **(c-d)** MMP-2 and MMP-9 levels were detected by western blot, and the relative protein expression was shown in histogram normalized to β-actin. **(e-f)** Validation of the relationship between PVT1 and the related protein levels of cell proliferation, migration and invasion through GSE76633 dataset. *P < 0.05, **P < 0.01, ***P < 0.001. Error bars indicate mean ± SD. (PDF 258 kb)

Additional file 5: **Table S3.** Predicted microRNAs binding to PVT1 3’UTR by bioinformatics analysis on DIANA. (DOCX 27 kb)

Additional file 6: **Table S4.** The differentially expressed miRNAs in GSE104165. (DOC 432 kb)

Additional file 7: **Figure S3.** Top 10 downregulated miRNAs in GSE104165 cohort. (PDF 193 kb)

Additional file 8: **Figure S4.** RIP assay confirmed that miR-143 was a target of PVT1. (**a-b**) The correlation among PVT1, miR-143 and Ago2 was determined by analyzing GBC-SD and NOZ cell lysates utilizing RIP with an Ago2 antibody. (**c-d**) qPCR was performed to detect the PVT1 level in the substrate of RIP assay in miR-143-overexpressing GBC cells. (**e**) Detection of PVT1 using qPCR in the sample pulled down by biotinylated PVT1 and negative control (NC) probe. (**f**) Detection of miR-143 using qPCR in the same sample pulled down by biotinylated PVT1 and NC probe. Input was used for normalization. *P < 0.05, **P < 0.01, ***P < 0.001. Error bars indicate mean ± SD (PDF 182 kb)

Additional file 9: **Figure S5.** The levels of PVT1 in GBC-SD and NOZ cell lines after transfection with lenti-sh-PVT1 or lenti-PVT1 and their corresponding control. (**a**) The PVT1 expression was significantly decreased in both GBC-SD and NOZ cell lines after transfection with lenti-sh-PVT1. (**b**) The PVT1 expression was significantly increased in GBC-SD cells after transfection with lenti-PVT1.*P < 0.05, **P < 0.01, ***P < 0.001. Error bars indicate mean ± SD. (PDF 146 kb)

The article "Long non-coding RNA PVT1 promotes tumor progression by regulating the miR-143/HK2 axis in gallbladder cancer" was retracted in 2025. Reasons: duplicated data; duplicate publication; overlap with earlier publications; unreliable data.

## Abbreviations

ceRNA: Competing endogenous RNA
GBC: Gallbladder cancer
HK2: Hexokinase 2
IHC: Immunohistochemistry
ISH: In situ hybridization
lncRNA: Long non-coding RNA
PVT1: Plasmacytoma variant translocation 1
qPCR: Quantitative real-time PCR
